# Deep Learning Approach for Discovery of In Silico Drugs for Combating COVID-19

**DOI:** 10.1155/2021/6668985

**Published:** 2021-07-20

**Authors:** Nishant Jha, Deepak Prashar, Mamoon Rashid, Mohammad Shafiq, Razaullah Khan, Catalin I. Pruncu, Shams Tabrez Siddiqui, M. Saravana Kumar

**Affiliations:** ^1^School of Computer Science & Engineering, Lovely Professional University, Phagwara, India; ^2^Department of Computer Engineering, Faculty of Science and Technology, Vishwakarma University, Pune, India; ^3^Cyberspace Institute of Advanced Technology, GuangZhou University, Guangzhou, China; ^4^Department of Engineering Management, University of Engineering and Applied Sciences, Swat 19060, Pakistan; ^5^Design,Manufacturing & Engineering Management, University of Strathclyde, Glasgow G1 1XJ, UK; ^6^Mechanical Engineering, Imperial College London, Exhibition Road South Kensington, London, UK; ^7^College of Computer Science and Information Technology, Jazan University, Jazan, Saudi Arabia; ^8^Department of Mechanical Engineering, Mount Zion College of Engineering and Technology, Pudukkottai, India

## Abstract

Early diagnosis of pandemic diseases such as COVID-19 can prove beneficial in dealing with difficult situations and helping radiologists and other experts manage staffing more effectively. The application of deep learning techniques for genetics, microscopy, and drug discovery has created a global impact. It can enhance and speed up the process of medical research and development of vaccines, which is required for pandemics such as COVID-19. However, current drugs such as remdesivir and clinical trials of other chemical compounds have not shown many impressive results. Therefore, it can take more time to provide effective treatment or drugs. In this paper, a deep learning approach based on logistic regression, SVM, Random Forest, and QSAR modeling is suggested. QSAR modeling is done to find the drug targets with protein interaction along with the calculation of binding affinities. Then deep learning models were used for training the molecular descriptor dataset for the robust discovery of drugs and feature extraction for combating COVID-19. Results have shown more significant binding affinities (greater than −18) for many molecules that can be used to block the multiplication of SARS-CoV-2, responsible for COVID-19.

## 1. Introduction

The first case of COVID-19 was detected in December 2019, and from then, it has overgrown, affecting millions of people around the globe. More than 2 million cases have been confirmed, with over 0.15 million deaths globally [1, 2]. Drug repurposing is defined as discovering and identifying newer applications for existing drugs in the treatment of various diseases [3]. Recent advancements in drug discovery using deep learning have made it possible to speed up identifying and developing new pharmaceuticals [4]. Various drugs, such as Arbidol, remdesivir, and favipiravir, have been tested to cure COVID-19 patients and many others are in the testing phase [4]. Biomedical researchers are investigating drugs for treating the patients, with an attempt to develop a vaccine for preventing the virus [5]. On the other hand, computer scientists have developed early detection models for COVID-19 from CT scans and X-ray images [5]. These techniques are a subset of deep learning and have been applied successfully in various fields [5]. Over the past few years, a significant increase in the quantity of biomedical data has resulted in the emergence of new technologies such as parallel synthesis and HTS (high-throughput screening), to mining large-scale chemical data [6]. Since COVID-19 is transmitted from person to person, electronic devices based on artificial intelligence may play a crucial role in preventing the spread of this virus. With the expansion of the role of health epidemiologists, the pervasiveness of electronic health data has also increased [7]. The increasing availability of electronic health data provides a massive opportunity for healthcare to enhance healthcare for both discoveries and practical applications [7]. For training machine learning algorithms, these data can be used to improve their decision-making in terms of disease prediction [7].

As the increase in the number of cases infected by coronavirus rapidly outnumbered the medical services available in hospitals, a significant burden on healthcare systems was imposed [7]. Because of the limited supply of hospital services and the delay in time for diagnostic test results, it is common for health professionals to provide patients with sufficient medical care. However, since the number of cases tested for coronavirus is growing increasingly day by day, testing is not feasible due to time and cost factors [7]. This paper aims at suggesting a technique based on deep learning which would be helpful in rapidly finding the drugs for combating the pandemic. Deep learning is currently an area that is quickly emerging and constantly expanding. To optimize its performance, it programs computers using data. Using the training data or its previous encounters, it learns the parameters to optimize the computer programs. It can also forecast the future using the data. Deep learning also lets us operate the statistics of the data to construct a mathematical model. The main goal of deep learning is that it learns without any human intervention from the feed data, and it automatically learns from the data (experience) provided and gives us the desired output where it searches the data trends/patterns [8]. Deep learning techniques have achieved greater efficiency in various tasks, including drug development, prediction of properties, and drug target forecasting. As drug development is a complex task, the deep learning approach makes this process faster and cheaper.

The challenges with COVID-19 at present make it necessary to look for some alternatives in medicine or drugs to combat the rise of cases due to COVID-19 infection. One of the significant challenges is the processing delay for the finalization of the drugs for vaccine formulation. However, many pharmaceuticals companies have achieved success to some extent after passing through different trials. Hence, predicting the most probable drugs for the vaccination formulation can speed up vaccine formulation and thus save many human lives. Another challenge is that most of the testing for vaccine formulation is done on a clinical basis where all the drug combinations are tried to get the desired selection of drugs. Still, there is less utilization of computational techniques for the same at present. Thus, there is an hour to look after some alternatives using some machine intelligence techniques to provide some solutions with more accuracy and at a faster note.

Based on the above challenges, the main contributions of the paper are as follows:

1. Deep learning approach based on logistic regression, SVM, and Random Forest along with QSAR modeling is proposed to discover some drugs for the treatment of COVID-19
2. QSAR modeling is done to find the drug targets with protein interaction along with the calculation of binding affinities
3. Deep learning models are used for training the molecular descriptors dataset for the robust discovery of drugs and feature extraction for combating COVID-19

The rest of the article is organized as follows.  Section 2 deals with the literature reviewed.  Section 3 deals with the significance of work.  Section 4 deals with the suggested methodology followed by Section 5, dealing with results, and the paper is concluded in Section 6.

## 2. Literature Review

Artificial intelligence techniques have been utilized in various areas of drug and vaccine development [9]. This utilization and further advancements are essential for immediately discovering a cure for the current pandemic. Many studies have been done previously, and many are ongoing to find a less complex and easy-to-use technique that would speed up the drug discovery process. In [10], the authors have trained a model based on LSTM (long short-term memory) for reading the SMILE fingerprints of a molecule for predicting IC50, binding to RdRp. The authors in [11] have suggested a B5G framework, which supports the diagnosis of COVID-19 through low latency and 5G. Choi et al. [12] proposed the MT-DTI model for predicting the drugs approved by FDA having solid affinities for the ACE2 receptor with TMPRSS2. The authors in [13] have reviewed all state-of-the-art research studies related to medical imaging and deep learning. Deep learning techniques and feature engineering were compared in order to efficiently diagnose COVID-19 from CT images [14]. Various neural network architectures and generative models such as RNN, autoencoders with adversarial learning, and reinforcement learning are suggested for ligand-based drug discovery [15]. Classification performance of DNN on imbalance compound datasets is explored by applying data balancing techniques in [16]. A novel approach for deep docking large numbers of molecular structures accurately is suggested in [17]. The effects of deep learning in drug design and complimentary tools were reviewed [18].

In [19], a systematic review of the application of deep learning techniques for predicting drug response in cancer cell lines has been done. A QSAR model (quantitative structure-activity relationship) is developed [20], which implements deep learning to predict antiplasmodial activity and cytotoxicity of untested compounds for screening malaria. In [21], the authors have built a multitask DNN model and compared the results with a single-task DNN model. In [22], various machine learning and deep learning algorithms used for drug discovery are reviewed, and their applications were discussed. However, various studies suggest deep learning for drug discovery or detecting COVID-19 lacks proper practical implementation with results. Most studies have just reviewed different deep learning techniques to be used for the development of drugs. This paper will give a practical implementation on various datasets available online with efficient results. Upon analyzing various studies, we found that various studies claim HCS (high content screening) as an efficient technique for screening chemical compounds for discovering drugs. At present, deep learning techniques have been producing faster and efficient results.

The basic idea of the screening process is that the cells are exposed to various compounds, and automated optical microscopy is done to see what happens, creating thriving images of cells. A quantitative and qualitative analysis of the result can be done by using an automated HCS pipeline. HCS branches out from microscopy, and Giuliano et al. first coined the terminology in the 1990s [23]. HCS research can cover several fields, such as discovering drugs that can be defined as a form of cell phenotypic screen. It includes methods of analysis that produce simultaneous readouts of multiple parameters considering cells or cell compounds. In this phase, the screening aspect is an early discovery stage in a series of various steps needed to identify new drugs. It acts as a filter to target potential applicants that can be used for further development. Small molecules classified as a low molecular weight organic compound, e.g., proteins, peptides, or antibodies, can be the substances used for this purpose [24].

## 3. Significance of the Work

Hospitals are using trial and error techniques for COVID-19 drug discovery [9]. It results in an emergence of virtual screening to discover chemical compounds due to the inefficiency of the lab-based HTS technique (high-throughput screening) [9]. Also, drug discovery and development is a complex and time-consuming process [25]. It is estimated that the preapproval cost of production of new drugs has increased at the rate of 8.5% annually from 802 million USD to 2870 million USD [26, 27]. Finding molecules with the required characteristics is one of the significant challenges in drug discovery. A practical and quality drug needs to be balanced regarding safety and potency against its target and other properties such as ADMET (Absorption, Distribution, Metabolism, Excretion, and Toxicity) and physicochemical properties [25]. This paper aims to increase the speed of discovering new molecules using deep learning, thereby reducing the cost of producing new drugs. Deep learning techniques will help us navigate large chemical spaces to find new chemical compounds [25]. The significance of using deep learning techniques for combating COVID-19 [1] is summarized in Table 1.

## 4. Suggested Methodology

This section includes a description of the proposed methodology.

### 4.1. Dataset Preparation and Preprocessing

We have used the combination of the datasets from the sources [29–31]. Each of the datasets contains a set of chemical compounds with respective binding activity to a target protein calculated by pIC50 *=* −log_10_(IC_50_) [32]. Preprocessing is done for removing the invalid and replicated compounds. The entries with IC50 measurements with filtered out compounds having suspicious measures are depicted by the “DATA VALIDITY COMMENT” column. For repeated records groups, if the standard deviation (SD) of the activity is found more significant than 1 log unit, then these datasets are deleted from the dataset, and a single entry is kept with the median of the activity [32]. Data preprocessing is one of the significant phases in data mining as it helps in achieving data integrity. Before preprocessing, data cleaning needs to be done as raw data contain abnormalities and errors affecting the results [33]. After preprocessing, conversion of SMILES [34] representations to molecular representations takes place. These are open datasets that contain the binding, ADMET, and functional information for various drugs like bioactive compounds [35]. The database containing the datasets has over 5 million bioactivity measurements for over 1 million compounds and over 5000 target proteins [35].

A minor challenge may occur in data mining algorithms due to variation in range and distribution of every variable in the large datasets due to distance measurements; also, these may contain noisy variables, which makes the learning of the algorithms more difficult [33]. These challenges can be handled by min-max normalization where the value of each variable is adjusted in a uniform range of 0 to 1 [33]. It is given in the following equation:

(1) $$\begin{array}{c} Y_{\text{normalised}}=\frac{Y_{x}-Y_{\text{minimum}}}{Y_{\text{maximum}}-Y_{\text{minimum}}}, \end{array}$$

where *Y*_normalised_ is the normalised value, *Y*_*x*_ is the value of interest, *Y*_minimum_ is the minimum value, and *Y*_maximum_ is the maximum value.

Apart from the dataset, the system used for performing the experiments has UBUNTU 20.04 LTS OS installed with 16 GB RAM and Intel Core i7-8700 processor. The language used for building the model is Python 3.7 with NumPy, pandas, TensorFlow, Bunch, tqdm, Matplotlib, scikit-learn, NVIDIA GPU, CUDA 9.0, Pytorch 0.4.1, Mordred, and RDkit. For evaluating the binding affinities, PyRx is used. We have used the regression model and QSAR techniques as regression models help us define relationships between dependent and independent variables and show the strength of the impact of various independent variables on dependent variables. QSAR helps in maintaining the quantitative structural relationships in molecular predictions.

### 4.2. Model Development and Evaluation Parameters

As mentioned above, developing a QSAR model can help us in defining the relationship between the chemical structures and their endpoints by using various statistical methods for the construction of predictive models for revealing the origin of bioactivity [36]. Generally, a QSAR model is depicted by the equation of the form *X*=*m*(*X*)+Err that can be utilized or prediction of endpoints or new compounds in terms of time-consuming and cost approaches. In order to derive the global molecular features for the SMILES, some notations are there [36], which are given in the following equation:

(2) $$\begin{array}{c} pqrstu\to p+q+r+s+t+u\left(X_{m}\right),\\ pqrstu\to pq+qr+rs+st+tu\left(XX_{m}\right),\\ pqrst\to pqr+qrs+rst+stu\left(XXX_{m}\right). \end{array}$$

Also, these global descriptors are described as follows [36]:

1. BOND is defined as the presence or absence of double (=), triple (#), and stereochemical (@) bond in SMILES
2. PAIR is defined as the coincidence of I, N, O, P, S, Br, Cl, F, #, @, and =
3. NOSP is defined as the presence or absence of P, S, O, and N
4. HALO is defined as the presence and absence of halogens

The optimal attributes for the SMILES are calculated by the following equation [36]:

(3) $$\begin{array}{c} W\left(X_{\text{epoch}},\text{Threshold}\right)==\sum TW\left(Xm\right)+\sum TW\left(XXm\right)+\sum TW\left(XXXm\right)+\sum TW\left(\text{NOSP}\right)+\sum TW\left(\text{BOND}\right)+\sum TW\left(\text{HALO}\right)\sum TW\left(\text{PAIR}\right). \end{array}$$

The chemical endpoints [36] can be given in the following equation:

(4) $$\begin{array}{c} \text{End}=T_{0}+T_{1}\times W\left(X_{\text{epoch}},\text{Threshold}\right), \end{array}$$

where *T*_*0*_ is the intercept and *T*_*1*_ is the correlation coefficient.

The development of the QSAR model consists of two significant steps: (i) describing the molecular structure and (ii) the multivariate analysis for correlation of molecular descriptors with observable characteristics [33]. Successful development of the model also includes data preprocessing and statistical evaluations. For evaluating the performance of the QSAR model, the statistical method suggested in [33] is used in the following equation:

(5) $$\begin{array}{c} x^{2}>0.5,\\ Y^{2}>0.6,\\ \frac{Y^{2}-Y_{0}^{2}}{Y^{2}}<0.1,\\ \text{or }\frac{Y^{2}-Y_{0}^{\prime \prime 2}}{Y^{2}}<0.1,\\ 0.85\leq z\leq 1.15\text{,}\\ \text{or }0.85\leq z^{\prime \prime }a\leq 1.15, \end{array}$$

where *x*^2^ is the cross-validated explained variance, *Y*^2^ is the coefficient of determination, *Y*_0_^2^ and *Y*_0_^″2^ are the predicted vs. observed activities and vice versa, respectively, and *x*^2^ is calculated by the following equation:

(6) $$\begin{array}{c} X^{2}=\frac{\sum_{j=1}^{\text{training}}\left(P_{j}-\hat{P_{j}}\right)2}{\sum_{j=1}^{\text{training}}\left(P_{j}-\hat{P}\right)2}, \end{array}$$

where *P*_*j*_ are the measured values, $\hat{P_{j}}$ are the predicted values, and *P*_*j*_ is the mean value of the entire dataset. This equation is also used for the calculation of external *x*^2^, i.e., the compounds that are not used in the QSAR model development earlier and are given in the following equation:

(7) $$\begin{array}{c} X_{{\text{external}}^{2}}=1-\frac{\sum_{j=1}^{\text{training}}\left(P_{j}-\hat{P_{j}}\right)2}{\sum_{j=1}^{\text{training}}\left(P_{j}-\hat{P_{j}}\right)2}. \end{array}$$

For measuring the internal chemical diversity [28], let *x* and *y* be two molecules having *Z*_*X*_ and *Z*_*Y*_ as their Morgan fingerprints [28]. The number of common fingerprints is defined as *Z*_*x*_∩*Z*_*y*_∨ and the total number of fingerprints is defined as *Z*_*x*_ ∪ *Z*_*y*_∨. The Tanimoto similarity [28] between *x* and *y* is defined in the following equation:

(8) $$\begin{array}{c} S\left(x,y\right)=\left|\frac{Z_{x}\cap Z_{y}}{Z_{x}\cup Z_{y}}\right|. \end{array}$$

And the Tanimoto distance [28] is given by

(9) $$\begin{array}{c} S_{d}\left(x,y\right)=1-S\left(x,y\right). \end{array}$$

We have used RDKit [28] for the implementation of Tanimoto distance. In earlier studies, the QSAR models were developed for small compounds that used limited quantitative characteristics [32]. Various algorithms were suggested for covering significant features, including hundreds or thousands of molecular descriptors. We have used the OPLRAreg algorithm suggested in [32] to illustrate the flexibility of mathematical modeling and show how the division of characteristics and regions helps enhance the features of OSAR datasets. The OPLRAreg is given in Algorithm 1.

Due to advancements in deep learning techniques, there has been an increase in the use of neural networks in a variety of applications including healthcare [25]. A neural network can be defined as a group of layers consisting of perceptrons called multilayer perceptron (MLP) or simply a neuron [25]. The perceptrons are the main building blocks of a perceptron and consist of three parts, weights, *v*=[*v*_1_, *v*_2_ … …, *v*_*n*_], *v*_*j*_ ∈ *R*, biases, *b* ∈ *R*, and an activation function, *f*(*n*) [25]. Let the input vector given to a perceptron be defined as, *x*=[*x*_1_, *x*_2_......, *x*_*n*_]^Q^. Then, the output is given in the following equation:

(10) $$\begin{array}{c} f\left(vx+b\right)=f. \end{array}$$

Both *v* and *x* should be in the same direction. Furthermore, for enabling the matrix multiplication, *b* and *x*_1_ should be appended to the weight and input vector, respectively [25] so that *v*=[*v*_1_*v*_2_ … *v*_*n*_*b*] and *x*=[*x*_1_*x*_2_ … *x*_*n*_1]^*Q*^.

And the output is given by

(11) $$\begin{array}{c} f\left(vx\right)=f\left(v_{1}x_{1}+v_{2}x_{2}+\cdots +v_{n}x_{n}+b\right). \end{array}$$

Due to an increase in the efficiency of computation, matrix multiplication is required for training larger networks with forward passing and backpropagation for optimizing the network parameters [25]. The different types of classification methods are given in the following sections.

#### 4.2.1. Logistic Regression

Logistic regression is the most used method of modeling for the prediction of risk [37]. A logistic regression model uses a role to render the model range output between zero and one and should therefore be used for classification. The logistic function is defined in [37] as follows:

(12) $$\begin{array}{c} Y\left(x=1\right)=\frac{1}{1+\exp-\left(\alpha r+s\right)}, \end{array}$$

where *r* is the input and *α* and *s* are called as model parameters. The output given is the modeled probability of the input belonging to a class [37]. For interpreting the meaning of the weights, rearrange the above equation as follows [37]:

(13) $$\begin{array}{c} \text{log}\left(\right)\log\left(\right)\alpha r+s. \end{array}$$

*Y*(*x*=1)/*Y*(*x*=0) is called as the odds. The modeling of odds is done through a linear equation [37]. Like most of the ML (machine learning) models, optimization of the parameters is done w.r.t. loss function [37]. Consider a given set of data points {(*p*_*j*_, *q*_*j*_)}_*j*_, where *p*_*j*_ is defined as the input and *q*_*j*_ is the true output. Let $\hat{q_{j}}$ denote the output of the logistic regressor. Then *α*∧*s* are selected according to [37] in the following equation:

(14) $$\begin{array}{c} \alpha^{*},\\ s^{*}{\text{argmin}}_{\alpha s}. \end{array}$$

This is also known as the log-loss function. The problem of minimization is solved iteratively until the convergence of parameters, using a coordinate descent algorithm [37].

#### 4.2.2. Random Forest

Random Forest is an ensemble approach that combines several decision trees to make predictions. More reliable and precise predictions can be made by combining several poor learners. In addition, ensemble techniques decrease variance and are less vulnerable to overfitting [37]. The Random Forest algorithm [38] is given in Algorithm 2.

As a sequence of questions, a decision tree is best defined. The principle is that questions are asked, and new questions are asked based on the responses, thus creating a tree. Data points are identified using the leaf nodes in the tree [37] by following the trajectory of the questions and answers. The tree is designed by determining which question to ask at each node and determined based on the information obtained from each possible query or the degree to which the uncertainty in the dataset [37] is reduced. The uncertainty in the dataset [37] is defined in the following equation:

(15) $$\begin{array}{c} \text{Entropy}\left(X\right)=-\sum_{\left|Xz\left\|\right)X\right|}y\left(X\right)\log_{2}\;y\left(X\right). \end{array}$$

The information is acquired by knowing the value of certain feature *F* and is given in the following equation:

(16) $$\begin{array}{c} \text{Gain}\left(F\right)=\text{Entropy}\left(X\right)-\sum_{z\in \text{values}}\frac{\left|\;Xz\right|}{\left|\;X\;\right|}\text{Entropy}\left(X_{z}\right), \end{array}$$

where *X*_*z*_ is defined as the subset where the feature *F* takes *z* value. Therefore, during the construction of a decision tree, a feature is to decide each node as explained in [37]. Here, the construction is either terminated once the entropy of the subset has reached zero or the tree has reached its maximum depth [37]. Upon evaluation of a sample, the tree's trajectory is decided until the leaf node is reached. An approximate probability can also be given as output by comparing the class sizes found in the leaf node [37].

#### 4.2.3. Support Vector Machine (SVM)

The support vector machine (SVM) is an algorithm for classification that involves creating a hyperplane. A set of features is used in order to classify an object. Thus, the hyperplane will lie in *p*-dimensional space if there are *p* features [39]. The hyperplane is generated through SVM optimization, which in turn maximizes the distance from the nearest points, also known as support vectors [39]. Let *y*_*j*_=[*y*_*j*1_,…,*y*_*jm*_]^*N*^ be an arbitrary observation feature vector in the training set, $\underline{x_{j}}$ corresponding label to *y*_*j*_, with a weight vector *v*=[*v*_1_,……,*v*_*q*_]^*N*^ with ∨*v*∨^2^=1 and *T* be the threshold. The constraints defined for the classification problem [39] are given in equations (17) to (20):

(17) $$\begin{array}{c} vNy_{j}+T>0\text{ for }\underline{x_{j}}=+1, \end{array}$$

(18) $$\begin{array}{c} vNy_{j}+T<0\text{ for }\underline{x_{j}}=-1. \end{array}$$

Let *f*(*y*_*j*_)=*V*^*N*^*Y*_*j*_+*T*, then the output of the model $\hat{x_{j}}$ can be given as follows:

(19) $$\begin{array}{c} \hat{x_{j}}=\left\{1\text{ for }f\left(y_{j}\right)\geq 0\right),\\ \left\{0\text{ for }f\left(y_{j}\right)<0\right). \end{array}$$

Instead of using ‖*v*‖^2^ = 1, for margin maximization, the lower bound on the margin along with the optimization problem can be defined for minimization of ‖*v*‖^2^ [39]. The constraints for the optimization problem can be derived from equations (17) and (18), respectively, [39] as follows:

(20) $$\begin{array}{c} \hat{x_{j}}vNy_{j}+T\geq 1. \end{array}$$

In some of the cases, it is required to implement a soft margin, allowing some points to lie on the wrong side of the hyperplane [39] in order to provide an efficient model. A cost parameter *M* is introduced, which plays a major role in the assignment of penalties to errors, where *M* > 0 [39]. Then, the minimized objective function [39] is defined as follows:

(21) $$\begin{array}{c} \vee v\vee 2+M\sum_{j}\beta_{j}, \end{array}$$

where *β*_*j*_=slack variable. The constraints to the optimization problems [39] are now modified in the following equation:

(22) $$\begin{array}{c} \underline{x_{j}}Ny_{j}+T\geq 1-\beta_{j},\;\beta_{j}\geq 0. \end{array}$$

Most of the datasets are not linearly separable. But through a nonlinear transformation into a high-dimensional space, a dataset is more likely to be linearly separable [37]. Therefore, each sample is transformed using a nonlinear function [37] so that

(23) $$\begin{array}{c} f:R^{X}⟶R^{Y},\;x>y. \end{array}$$

And then the problem is considered using *m*_*j*_=*f*(*y*_*j*_) [37]. Furthermore, using Lagrange optimization, the dual problem of maximizing [37] is defined as follows:

(24) $$\begin{array}{c} \sum_{j}\left[\delta_{j}-\frac{1}{2}\underset{i}{\sum }\delta_{j}\delta_{i}T_{j}T_{i}\lambda y_{i}\right],\;\lambda =yjt, \end{array}$$

subject to the condition

(25) $$\begin{array}{c} \sum_{j}\delta_{j}T_{j}=0,\;\delta_{j}\geq 0\forall j. \end{array}$$

The overall structure of the workflow and QSAR modeling [36, 40] is explained in Figure 1. First, we have to select the number of molecules. It can be of any number. Each molecule has its molecular descriptors that describe the molecules' physical and chemical properties that help us differentiate between the molecules. Here, 1 and 0 are the binary descriptors that show the presence/absence of the molecular descriptors. A collection of these descriptors constitutes the dataset. Values of *X* (active/inactive) show the biological activity we want to predict. This dataset is now used for training the deep learning model, which therefore gives our results. The working of the proposed approach is represented in a flowchart, as depicted in Figure 2.

## 5. Results

Our goal is to develop a deep learning model to suggest novel and effective drugs for combating SARS-CoV-2 or combating COVID-19. Our regression-based models and Random Forest model were trained on a dataset of approximately 1.5 million drug-like molecules from the data sources [29–31]. The molecules were represented in Simplified Molecular Input Line Entry System (SMILES) format helping our model learn the required features for designing novel drug-like molecules. SMILES are defined as the character strings for representing drug molecules. For example, an atom of carbon can be represented as C, oxygen atom as O, double bond as =, and CO_2_ molecule can be represented as C(=O)=O. The maximum length of the string can be taken as 25 [41]. SMILES grammar's learning problem and reproducing it for generating novel small molecules is considered a classification problem [42]. The SMILES strings should be considered a time series, where every symbol is considered a time point. At a given point, the model was trained for predicting the class of the next symbols in the time series.

We will only retrieve the coronavirus proteinase during preprocessing of the bioactivity data that can be reported as IC50 values in nM (nanomolar) units [43]. The data for bioactivity is in the IC50 unit. Compounds with less than 1000 nM values will be considered active, whereas compounds with values greater than 10,000 nM will be considered inactive. As for such values, the intermediate value is between 1,000 and 10,000 nM [43]. To evaluate the model, Lipinski descriptors [43] were used as given in Table 2.

Upon analyzing the pIC50 values, the actives and inactives have shown a significant difference, which is expected as the values of IC  < 1000nM = active, IC50 > 10000nM = inactive, corresponding to pIC50 >6 = active and pIC50  <5  = inactive. Out of the 4 Lipinski descriptors [43], only log*P* showed no difference between the actives and inactives, while the other three descriptors showed significant differences between the actives and inactives. This can be better understood by Figures 3–7 , respectively. A scatter plot has also been drawn to show that the two bioactivity classes (active/inactive) are spanning similar chemical spaces.

Figures 3–7 show that our model can explore the chemical spaces that are further adapted for generating the smaller molecules specific to a target of interest. The SARS-CoV-2 contains the proteins responsible for the cation and replication of the virus [44]. The functioning of the proteins can be stopped by introducing the drug molecules capable of blocking the protein. Therefore, we have to find the molecules with a high binding affinity to bind the protein effectively. Various drugs/compounds have been tested for finding a high binding relationship, but the results are not very good. We have created novel molecules for binding with the coronavirus, using deep learning and QSAR modeling. After the generation of the molecules, PyRx was used for evaluating the binding affinities. We have also build a regression model using a Random Forest algorithm for acetylcholinesterase inhibitors, as shown in Figure 8. The binding affinities for leading drugs for other diseases such as HIV inhibitors range from −10 to −11. Also, the most recent drug remdesivir, which is clinically tested, has the binding affinity of −13. By convention, the more negative the scores are, the more effective the drugs would be. QSAR modeling, docking analysis, and use of regression model generate a list of bioactive compounds from which top 100 compounds were selected, which may have the potential to be effective against SARS-CoV-2. The methodology suggested in this paper is easy to use and can be a possible technique for the discovery of anti-COVID-19 drugs and also shortening the clinical development period required for drug repositioning. Our proposed methodology can give the binding affinity more than the present drugs being tested, making our approach efficient. The proposed list of top 100 chemical structures or molecules generated using our proposed approach through SMILES software is shown in Table 3.

## 6. Conclusion

Drug development is a time-consuming and expensive process. Deep learning has achieved excellent performance in a lot of tasks. Drug discovery is one of the areas that can be benefitted from this. The use of deep learning techniques has made the process of drug development more manageable and cheaper. Deep learning-based models can learn the feature representations based on present drugs that can be used to explore the chemical spaces in search of more drug-like molecules. The available data for automating the processes and better predictions are what deep learning techniques promise for efficient drug discovery. These techniques have proven effective in scanning peptides or detecting COVID-19 from the CT scan or X-ray images. These techniques can speed up the drug development process but require clinical testing for more validation and accuracy [45].

## Figures and Tables

**Figure 1:** Overall workflow of the suggested methodology.

**Figure 2:** Flowchart depicting the complete working of the proposed approach.

**Figure 3:** Scatter plot of MW vs. log*P*.

**Figure 4:** Box plot of MW.

**Figure 5:** Box plot of log*P*.

**Figure 6:** Box plot of NumH donors.

**Figure 7:** Box plot of NumH acceptors.

**Figure 8:** Scatter plot for experimental vs. predicted values of pIC50 for regression model developed for acetylcholinesterase inhibitors.

**Algorithm 1:** OPLRAreg algorithm.

**Algorithm 2:** Random Forest algorithm.

**Table 1:** Summary of applications of deep learning for combating COVID-19.

S. no.	Application	Explanation
1	Pandemic tracking [1]	(i) Bidirectional GRU along with attentional techniques are used for analyzing patterns in respiratory images for mass scale screening of COVID-19 (ii) Application of deep learning (DL) techniques for identification of geographical hazards and spreading at the community level
2	Predicting the structure of proteins [2]	(i) CNN, DNN, and deep ResNet architecture are utilized for the identification of characteristics of proteins (ii) Virus-host prediction and early prevention of virus infectivity can be done using DL architectures
3.	Drug discovery [25]	(i) GAN and reinforcement learning techniques should be implemented for discovering the chemical compounds inhibiting COVID-19
4.	Medical imaging[28]	(i) DL architecture should be used for extraction of features and prediction of possible cases of COVID-19 from CT scan or chest X-ray images

**Table 2:** Calculated values of Lipinski descriptors.

MW	Log*P*	NumH donors	NumH acceptors
281.3	1.90	0.0	5.0
416.5	3.82	0.0	2.0
422.2	2.67	0.0	3.0
294.3	3.63	0.0	4.0
339.3	3.54	0.0	5.0
338.4	3.41	0.0	5.0
297.0	3.45	0.0	3.0
277.2	4.10	0.0	3.0
278.3	3.30	0.0	3.0
282.4	4.11	0.0	2.0

**Table 3:** Top 100 compounds generated using the proposed approach.

Serial no. of the chemical structure generated	SMILES generated chemical structure generated through the proposed approach	Binding affinity value (kcal/mol)
1	Cc1ccc(C2CNCCN2C)cc1	−23.1
2	CCOC(CO)c1ccccc1	−15.2
3	CC(=O)Nc1cnn(C)n1	−24.6
4	CCC(C)NCc1ncccn1	−21.5
5	CC(C)=C1CC(N)C1	−20.4
6	CN1CCCc2cc(CON)ccc21	−18.9
7	CC12CNCC1CN(CC(N)=O)C2	−28.9
8	CCNC(C)C(C)c1cnccc1C	−19.5
9	CCN(Cc1ccccc1)C(C)CCCNC	−18.1
10	CCC(=O)c1cc(C)ccn1	−18.3
11	C=CC(O)c1cc(C)ccn1	−21.5
12	C#CCCOc1cnccc1C	−16.8
13	Cn1nc2ccccc2c1S(N)(=O)=O	−19.8
14	Cn1cnn(CC(N)=O)c1=O	−23.1
15	CC(NCCSc1ccccc1)c1ccncc1	−21.6
16	Cc1ccsc1-c1ccc(O)nc1	−21.9
17	N#Cc1ncccc1N1CC2CC1CN2	−19.6
18	N#Cc1cnccc1SCC(N)=O	−23.6
19	N#Cc1ccc(C2NCCCCC2=O)cn1	−23.5
20	CC(C)C(C)Sc1ccc(C#N)cn1	−18.6
21	Cc1ccnc(C=CCCN)c1	−24.2
22	CCOC(CC)C(=O)c1cnccc1C	−15.9
23	Cc1ccncc1C(O)CNCC(C)C	−22.2
24	CS(=O)(=O)c1ncc(N)cn1	−21.1
25	OCC(O)CCSCc1ccccc1	−19.8
26	COC(=O)CNCc1cc(C)ccn1	−19.5
27	CCOC(c1ccccc1)C(CC)NN	−18.0
28	Cc1ccncc1C(=O)CCCN(C)C	−19.3
29	C=CCCSCCNc1cc(C)ccn1	−21.2
30	CCNC(=S)NNC(=O)Cc1ccccc1	−23.6
31	OC(CCCc1ccccc1)c1cccnc1	−20.4
32	CC(=O)CC(C)c1cnccc1C	−17.3
33	CN1CCC(O)(c2ccoc2)CC1	−18.1
34	Cc1ccnc(NC(=O)C#CCN)c1	−24.1
35	N#Cc1cnccc1NCCCO	−21.0
36	CCSCc1cncc(C#N)c1	−19.4
37	NC1=CCOC1=O	−16.4
38	CNC(CSC1CCCCC1)Cc1cccnc1	−18.7
39	COC(=O)c1ccc(C(C)C=O)cc1	−14.3
40	CC(=O)CC(O)c1cnccc1C	−21.0
41	CCCNCc1ccccc1S(N)(=O)=O	−20.8
42	N#Cc1nccnc1N1CCCOCC1	−22.0
43	CCC(CC)Oc1ncccc1C#N	−16.8
44	CC(C)(C)C(C)(N)c1ccccc1	−17.0
45	CN(C)NCc1ccccc1	−20.0
46	NC12CCCC1CNC2	−24.3
47	C(=Cc1ccccc1)CNCc1cccnc1	−23.8
48	CCNCCNc1ncccc1C#N	−26.6
49	CC(C)OCc1ccc(C#N)cn1	−18.3
50	NC1Cc2csnc2C1	−26.5
51	Cc1ccsc1C1NCCCCC1O	−21.3
52	N#CCCNCc1cncnc1	−20.8
53	COC(=O)c1ccccc1C#CCO	−15.5
54	N#CC1CN(CCN)C(=O)O1	−19.4
55	CC(CCO)Nc1ccc(C#N)cn1	−22.6
56	NC1CC2(CCNC2=O)C1	−21.8
57	C#CC(CO)NCc1cnccc1C	−22.6
58	CN1CCCc2cccc(OCC#N)c21	−16.2
59	NNC(c1ccncc1)C1CCCCC1	−23.8
60	C#CCCSc1ncccn1	−17.2
61	Cc1ccncc1C(C)(N)C(C)C	−22.6
62	NS(=O) (=O)c1ccc(SCCO)cc1	−21.0
63	Cc1ccnc(CC(=O)C(=O)O)c1	−18.8
64	CN1CC2CCN(CC(N)=O)C2C1	−25.9
65	O=C=NCc1ccncn1	−20.9
66	Cc1cscc1C1CC(O)CN1	−19.2
67	O=C(CC1CCCCC1)NC1CCCNCC1	−22.4
68	CC(O)Cc1cncnc1	−20.8
69	CCC(CC)Oc1ccc(C#N)cn1	−16.1
70	Cc1ccnc(NN=CC(C)C)c1	−19.7
71	COC(CNCCCOCc1ccccc1)OC	−12.3
72	N#Cc1ncccc1C1CCCCC1	−18.3
73	NC1COC2COCC12	−19.9
74	COC(=O)c1ccccc1C=CCCO	−18.6
75	CCCC(C)Sc1ncccn1	−16.9
76	CC(C)CC(=O)NCCCc1ccccc1	−16.8
77	CCC(CC#N)Nc1ccc(C#N)cn1	−21.8
78	CCCC(C)C(=O)c1cc(C)ccn1	−19.0
79	CCOc1cncnc1	−18.6
80	NCCCCC(O)c1ccccc1	−21.0
81	N#CCNc1ccncc1C#N	−21.6
82	N#Cc1cnccc1NCC=CCN	−27.2
83	CCCOCC(NC)c1cc(C)ccn1	−18.6
84	Nc1ccc(S(N)(=O)=O)cc1	−22.4
85	c1cncc(OCCNC2CCCCC2)c1	−20.8
86	CSCC(C)CNc1ncccc1C#N	−21.1
87	CC(N)CNc1cncnc1	−26.8
88	CC(C)(N)CNC(=O)Cc1ccccc1	−22.2
89	NC(CO)c1ccncn1	−26.9
90	CC(=O)OCSc1ncccn1	−19.3
91	CN1CCCc2cccc(C=O)c21	−16.4
92	CCNc1cc(NCC(C)(C)O)ccn1	−25.6
93	CCC(CC)CC(=O)COCc1ccccc1	−13.0
94	C=CCCC(=O)OCc1ccccc1	−13.9
95	CN(CCCO)C(=O)Oc1ccccc1	−18.8
96	CSCCC(=O)c1cncnc1	−19.6
97	CC(C)CCCC(O)CCOCc1ccccc1	−13.9
98	COc1ccncc1C#N	−18.1
99	CNc1nc(N)ncc1N	−28.4
100	c1ccc(CONCCNc2ccncc2)cc1	−25.4

## Data Availability

The data used to support the findings of this study are available from the corresponding author upon request.
